# The Value of Emergency Nursing Mode in the Treatment of Patients with Traumatic Shock

**DOI:** 10.1155/2022/6887236

**Published:** 2022-01-06

**Authors:** Jinmei Xu, Xueying Zhou, Chunying Wang, Jianli Hu

**Affiliations:** ^1^Ningbo College of Health Sciences, Ningbo 315104, China; ^2^Ningbo Mingzhou Hospital, Ningbo 315104, China; ^3^Hwa Mei Hospital, University of Chinese Academy of Sciences Department of Nursing, Ningbo 315104, China; ^4^The Affiliated Hospital of Medical School of Ningbo University, Ningbo 315104, China

## Abstract

**Objective:**

To study the value of emergency nursing mode in patients with traumatic shock.

**Methods:**

76 patients with traumatic shock in our hospital from March 2019 to February 2021 were selected and divided into study group and control group according to different rescue modes, 38 cases in each group. The study group adopted emergency nursing mode for rescue, while the control group adopted routine nursing mode for rescue. The rescue intervention, emergency stay and preoperative preparation time, rescue success rate, emergency rescue effect, complications, and satisfaction rate of patients and their families for rescue were compared between the two groups.

**Results:**

The rescue intervention, emergency stay and preoperative preparation time of the study group were significantly shorter than those of the control group, and the difference was statistically significant (*P* < 0.05). The rescue success rate of the study group was 97.37%, which was significantly higher than 84.21% of the control group, and the difference was statistically significant (*P* < 0.05). The improvement rate of the study group was significantly higher than that of the control group, the disability rate was significantly lower than that of the control group, the overall emergency rescue effect was better than that of the control group, and the difference was statistically significant (*P* < 0.05). The incidence of complications in the study group was 2.63%, which was significantly lower than 23.68% in the control group (*P* < 0.05). The satisfaction rate of patients and their families in the study group was 97.37%, which was significantly higher than 84.21% in the control group (*P* < 0.05).

**Conclusion:**

Emergency nursing mode in patients with traumatic shock owns higher rescue value, can buy time for the operation, improve the success rate and effect of rescue, make safety and satisfaction higher. Overall, for patients with traumatic shock, emergency nursing mode is better than conventional rescue nursing.

## 1. Introduction

Traumatic shock is due to the body suffered from violence, the occurrence of important organ injury, severe bleeding, and other conditions, resulting in a sharp reduction in effective circulating blood volume and insufficient perfusion of circulating tissue [1]. The incidence is closely related to the nature of the injured object, the site of injury, the degree of blood loss, the physiological condition, and the early treatment after injury. With the accelerating pace of modern life, the incidence of severe multiple injuries is increasing, among which the mortality of traumatic shock is the highest and the success rate of treatment is the lowest [2]. According to WHO statistics, about 10% of deaths and 16% of disabling cases worldwide are due to trauma and are also the leading cause of death in people under 40 years of age worldwide. Traumatic hemorrhagic shock accounts for more than 60,000 deaths each year in the United States and more than 1.5 million worldwide. Multiple organs of patients with severe trauma are seriously injured at the same time (or successively). The condition is complex and dangerous. In addition to the direct injury factors causing damage to the function of the affected organs, various pathological mechanisms often lead to damage to the function of other organs except the damaged organs. Traumatic shock is the main cause of death in emergency surgery due to its high mortality and disability rate and complicated diagnosis and treatment. Therefore, how to correctly assess the severity of traumatic shock patients, closely monitor the hemodynamic changes, and timely give effective fluid resuscitation become the key to successful treatment. There is insufficient effective circulating blood volume in the early stage of traumatic shock. If it is not treated in time, it can lead to insufficient perfusion of important tissues and organs, anaerobic metabolism, lactic acidosis, reperfusion injury, and endotoxin translocation, which will eventually lead to multiple organ failure and death. For emergency medical staff to respond quickly, we must immediately take emergency measures to improve the prognosis. Due to the rapid and complex changes in the condition of critically ill patients in the emergency department, the emergency time is urgent, the rescue task is heavy, and the medical staff are in a tense working state. The comprehensive professional quality and working mode of medical staff are very important for the emergency efficiency and the prognosis of patients. How to improve the quality of emergency care in the emergency department has been widely concerned. Scientific emergency rescue nursing mode is very important for the guarantee of patients' quality of life [3]. Therefore, 76 patients with traumatic shock who were hospitalized from March 2019 to February 2021 were studied to evaluate the value of emergency rescue nursing. The report is as follows [4].

## 2. Materials and Methods

### 2.1. Clinical Data

76 patients with traumatic shock who were treated in our hospital from March 2019 to February 2021 were selected as the research objects and divided into study group and control group according to different rescue modes, 38 cases in each group. There were 24 males and 14 females in the study group; age ranged from 17 to 65 years old, with an average age of 42.4 ± 4 years old; there were 6 cases of crush injury, 14 cases of falling injury, 13 cases of traffic accident injury, 3 cases of smashing injury, and 2 cases of penetrating injury in the injury type [5]. In the control group, there were 23 males and 15 females; age ranged from 17 to 64 years old, with an average age of 42.6 ± 5 years old, including 5 cases of crush injury, 15 cases of falling injury, 14 cases of traffic accident injury, 2 cases of smashing injury, and 2 cases of penetrating injury. There was no significant difference in gender, age, and other basic data of all patients (*P* > 0.05), which was comparable [6].

### 2.2. Inclusion Criteria and Exclusion Criteria

Inclusive criteria: (1) all patients met the diagnostic criteria of traumatic shock. (2) All patients were treated within 24 hours after injury. (3) The family members of the patients signed the informed consent to know and support the study. (4) No mental illness can cooperate with the treatment independently [7].

Exclusion criteria: (1) patients with heart, lung, and other important organ dysfunction. (2) Patients with unclear consciousness and unable to communicate normally.

### 2.3. Methods

In the control group, the traditional nursing mode was used, that is, the establishment of venous channel, infusion of dilatant fluid, and hemostasis treatment. Oxygen inhalation and trauma treatment were carried out in time. Vital signs were measured.

The study group applied the emergency nursing mode. ①To develop a perfect emergency process for patients with traumatic shock, establish an efficient and fast trauma emergency nursing team, select experienced emergency nurses as the team leader, actively lead nursing members to carry out the correct emergency nursing mode, and clarify the responsibilities and work norms of nurses [8]. After admission, the patients were evaluated comprehensively, all kinds of emergency situations were predicted, the ward and operating room were informed in advance, and the corresponding emergency measures were taken to open the green rescue channel [9]. Reduce the procedures of admission and triage and treat the patients as soon as possible. In the whole process of emergency rescue, medical staff are required to respond quickly, think clearly, act quickly and timely, strengthen the cooperation between departments, shorten the time of each handover link, and strive for the rescue time to the greatest extent. ② Attention should be paid to prehospital first aid, and publicity and training should be strengthened. The treatment of severe trauma should focus on keeping breathing unobstructed, hemostasis, limiting activities, fixing injured limbs, replenishing blood volume, and preventing hypovolemic shock. Make patients stay absolutely in bed, add bed baffle, and avoid falling into bed and other accidents [10]. The respiratory rhythm, heart rate, urine volume, blood pressure, and other indicators of the patients were closely monitored. The consciousness of the patients was observed, and whether the patients had symptoms such as cold limbs, pale face, fracture performance, apathy, and sweating were understood, so as to make correct treatment for the patients in time. ③ For targeted treatment of injury, we should first quickly understand the specific injury of patients, for the existence of organ injury, fracture patients, to timely surgery. Close observation of the condition, monitoring of vital signs, and early detection of shock symptoms. When the breathing is abnormal, the first aid plan of tracheal intubation and tracheotomy should be considered, and the whole process should be alert to ischemia and hypoxia. ④ Hemostasis and pain relief: quickly judge the bleeding site and adopt aseptic dressing, tourniquet, pressure bandage, and other programs. Abdominal puncture or peritoneal lavage should be performed as soon as possible in patients with closed abdominal injury or organ rupture. If the bleeding is not serious, the operation should be carried out after the blood volume is basically replenished and the shock is basically corrected. After the occurrence of traumatic hemorrhagic shock, the effective circulating blood volume will decrease, and then the adverse conditions such as blood pressure reduction, hypoxia, and kidney injury will appear [11]. The first step is to find out the cause and take hemostatic measures. The second step is to relieve pain effectively. The body's stress response increases under severe pain, and it will also increase the patient's negative emotion and body oxygen consumption. The shock symptoms will then worsen and become a vicious circle. ⑤ Keep breathing unobstructed and improve the state of hypoxia: most patients have respiratory disorders, tissue oxygen metabolism interference, and respiratory tract obstruction. The head of the patient was tilted to one side, and the secretions and blood clots in the oral cavity and nasal cavity of the patient were fully wiped with sterile gauze. If the patient is in a coma state, the tongue should be clamped outside the mouth with tongue clamps to avoid airway obstruction caused by tongue falling back. If necessary, the patients can be treated with endotracheal intubation and low flow oxygen inhalation [12]. Patients with dyspnea should be intubated according to the doctor's advice. When PaCO_2_ is more than or equal to 60 mmHg, a ventilator should be used. If necessary, the PaO_2_ of patients can be maintained at 70–100 mmHg. At the same time, the skin color, temperature, and humidity were observed. If the patient's skin is pale and cool, it means that he is in the period of microcirculation spasm [13]. During this period, the blood flow of the patients decreased significantly. If the patient has cyanosis of skin and mucous membrane and cold and wet limbs, it indicates that he is in the period of microcirculation expansion. During this period, the blood flow in the body of patients is relatively slow, and they have severe symptoms of hypoxia. If there are bleeding spots and ecchymosis on the chest and abdominal wall, it indicates that the patient is in the stage of disseminated intravascular coagulation. During this period, the blood in the patient was hypercoagulable. ⑥ Blood volume supplement: rapid establishment of venous channels for volume expansion. Early, rapid, and sufficient volume expansion is the key to successful rescue of shock. Intravenous indwelling puncture needle should be used to establish at least two venous channels for rapid and large-scale infusion and blood transfusion. The balanced solution should be given priority to, and crystal should be used before colloid to improve the insufficient circulating blood volume and correct acidosis. At the same time, venous blood was collected for blood type identification, cross matching, and blood preparation. Blood samples were taken from the patients and sent to the laboratory to test the corresponding indicators. The patients with lower blood pressure were given vasoactive drugs according to the doctor's advice. If venipuncture is difficult, deep vein catheterization is necessary, or phlebotomy and catheterization can be used. Depending on the amount and location of bleeding, the hemostasis operation was completed with sterile gauze pressure bandage, vascular forceps, tourniquet and silk thread ligation, and the hemostasis time was accurately recorded. At the same time, the tourniquet was opened once every half an hour to avoid limb necrosis [14]. If conditions permit, patients can be treated with debridement and hemostasis. If there is massive hemorrhage in the chest and abdominal cavity, antishock treatment should be given immediately [15]. Meanwhile, emergency operation should be taken to identify the focus and stop bleeding. The control group received routine emergency care, including opening airway, hemostasis, condition evaluation, and ensuring airway patency. ⑦ Prevention of infection and nutritional intervention: infection is very easy to occur in the early stage of trauma. In the process of first aid, debridement, cleaning, and anti-inflammation should be carried out to avoid the occurrence of wound infection [16]. Macrolide antibiotics and cephalosporins were used to control infection. When the nurses clean up the wound of the patients, for the patients with fracture, they should temporarily fix the fracture site according to the doctor's advice and then inform the orthopedic doctor to consult the patient's condition. ⑧ In addition to ensuring the rescue effect, the emergency nursing process model attracts more importance to the patient's psychology, patient's emotional changes, and family members' emotional changes and satisfaction and fully considers the needs of patients as social people. The traditional routine care process model may pay more attention to the effect of rescue and treat the patient as only a biological person [17].

### 2.4. Observation Indexes

#### 2.4.1. Emergency Intervention, Emergency Stay, and Preoperative Preparation Time

The rescue intervention, emergency stay, and preoperative preparation time of the two groups were statistically analyzed and compared.

#### 2.4.2. Rescue Success Rate

The number of successful rescue cases in the two groups was counted, and the success rate was compared.

#### 2.4.3. Emergency Rescue Effect

The improvement, stability, and disability of the two groups were compared.

#### 2.4.4. Complications

The complications such as disseminated intravascular coagulation, acute respiratory distress syndrome, and multiple organ dysfunction were compared between the two groups.

#### 2.4.5. The Satisfaction Rate of Patients and Their Families to Rescue

A self-made family satisfaction questionnaire was used to comprehensively assess the satisfaction of patients and their families with nursing. The satisfaction of patients and their families to the rescue was divided into very satisfied, relatively satisfied, and not very satisfied. The satisfaction rate was the percentage of very satisfied and relatively satisfied.

### 2.5. Statistical Methods

SPSS 26.0 software was used for data processing and analysis. Enumeration data were expressed as percentage (%), and *χ*^2^ test was performed. Measurement data were expressed as mean ± standard deviation ($\bar{x}\pm s$), and the data were compared by *t*-test. *P* < 0.05 as the difference was statistically significant.

## 3. Results

### 3.1. Emergency Intervention, Emergency Stay, and Preoperative Preparation Time

The rescue intervention, emergency stay, and preoperative preparation time of the study group were significantly shorter than those of the control group, and the difference was statistically significant (*P* < 0.05). See Table 1.

### 3.2. Rescue Success Rate

The rescue success rate of the study group was 97.37%, which was significantly higher than 84.21% of the control group, and the difference was statistically significant (*P* < 0.05). See Table 2.

### 3.3. Emergency Rescue Effect

The improvement rate of the study group was significantly higher than that of the control group, the disability rate was significantly lower than that of the control group, the overall emergency rescue effect was better than that of the control group, and the difference was statistically significant (*P* < 0.05). See Table 3.

Permanent disability refers to irreversible functional activity disorders caused by diseases or injuries, such as posttraumatic amputation and paralysis after complete spinal cord injury.

### 3.4. Complications

The incidence of complications in the study group was 2.63%, which was significantly lower than 23.68% in the control group (*P* < 0.05). See Table 4.

### 3.5. The Satisfaction Rate of Patients and Their Families to Rescue

The satisfaction rate of patients and their families in the study group was 97.37%, which was significantly higher than 84.21% in the control group (*P* < 0.05). See Table 5.

## 4. Discussion

Traumatic shock refers to the rapid decline of effective circulating blood volume in the body and the serious lack of blood perfusion in the tissue after severe trauma, which eventually leads to the body's important organs hypoxia, ischemia, and tissue cell metabolism disorders and other systemic pathological process [18]. Traumatic shock is one of the common surgical emergencies, which mostly occurs in young men. With the progress of society, city construction and high speed roads have also been developing rapidly. Incidence rate of traumatic shock has also increased year by year. Traumatic shock is the body's emergency response after trauma. Most of the patients are due to acute bleeding after fracture and organ injury. At the same time, toxic substances produced by tissue catabolism are also the cause of shock. If not treated in time, the life safety of patients will be seriously threatened. Therefore, taking correct and effective emergency measures as soon as possible has a positive impact on the success rate of rescue [19]. Traumatic shock in clinical treatment, is a common situation, in the implementation of timely and effective treatment process, should also cooperate with nursing intervention; in the past nursing, the common nursing method is the traditional routine nursing, although effective, but the effect is not satisfactory. In order to improve the quality of nursing, the emergency nursing mode was adopted. First aid nursing is a new type of nursing, and in the implementation process, patient evaluation should be first implemented, so that nursing staff can fully understand the actual condition of the patient and prepare for the follow-up care. Through the observation and nursing of patients' condition, prompt treatment and the life safety of patients can be guaranteed [20]. Through preoperative preparation, the patients' anxiety, depression, and other adverse emotional reactions can be improved, and thus, the satisfaction rate of patients and their families and the success rate of treatment can be improved to a certain extent [21].

To explore the value of emergency nursing mode in the rescue of traumatic shock patients, 76 patients with traumatic shock were selected for group study [22]. The results showed that the time of rescue and hospitalization of the patients in the observation group was significantly shorter than that of the control group, which was consistent with the reports of Yangzhihua and others. It suggested that the first aid nursing measures could effectively improve the success rate of the patients with traumatic shock. The reason is that rescue and nursing process implemented by the study group in this study is closely coordinated and the division of labor is clear in addition to skilled professional skills. The rescue work greatly reduces blindness and repetition due to the standardized rescue process, effectively avoids the waste of human resources, and obviously shortens the rescue time [23]. Therefore, the rescue success rate of the study group was significantly higher than that of the control group. Before implementing the emergency rescue nursing process, because of the lack of standardized work procedure, nurses often lack clear nursing objectives, and the rescue effect of patients is also different due to the difference of nurses' professional technology. The rescue and nursing process has fundamentally changed the above situation. Because of the formulation of the standard, nurses have been greatly strengthened in the operation skills and emergency ability of rescue. Nurses gradually changed from the original passive execution of medical orders to actively implement all rescue work, greatly reducing the waste of time in the rescue process and effectively improving the success rate of rescue. Other studies show that whether the patients with traumatic shock can survive depends on whether they can get effective emergency treatment in a short time [24].

Some studies have pointed out that the emergency nursing model has improved the requirements for nurses to a certain extent [25]. The nursing staff not only needs to have professional theoretical skills but also needs to have skilled operation ability and high sense of responsibility to treat and care for them in the shortest time, so as to reduce the incidence of complications. In addition, in the application process of emergency rescue nursing mode, nurses are also required to have keen ability, so as to observe the condition in time, so as to improve the success rate of treatment. In addition, in the application of emergency rescue nursing mode, we should fully cooperate with doctors, so as to achieve the smooth diagnosis and treatment process [26]. The results showed that the improvement rate of 69.23% in the experimental group was higher than that of 38.47% in the control group, and the disability rate of 0.00% was lower than that of 15.38% in the control group. The study concluded that the difference between the two groups was statistically significant. The stability rate of the two groups was compared (30.77% in the experimental group vs. 46.15% in the control group), and the difference was not statistically significant. The data confirmed that patients with traumatic hemorrhagic shock emergency care mode, in the fastest time to accept diagnosis and treatment, so that the success rate of rescue patients is higher. And, the rescue time of the experimental group was 45.72 ± 19.23 minutes, which was shorter than that of the control group (62.55 ± 20.02 minutes), and the difference was statistically significant; the incidence of complications in the experimental group was 7.69%, lower than 30.77% in the control group, and the difference was statistically significant [27, 28]. The emergency rescue and nursing model enhances the requirements of nursing staff to a certain extent. The nursing staff not only needs to have professional theoretical skills but also needs to have skilled operation ability and high sense of responsibility to treat and care for them in the shortest time, so as to reduce the incidence of complications [29].

In related studies, after the application of emergency nursing mode, the rescue intervention time, emergency stay time, and preoperative preparation time of the observation group were lower than those of the control group, the rescue success rate of the observation group was higher than that of the control group, the incidence of multiple organ dysfunction syndrome and asphyxia of the observation group was lower than that of the control group, and the satisfaction score of the family members of the observation group was higher than that of the control group. It shows that the emergency nursing mode has achieved the expected treatment effect in the nursing of patients with traumatic shock. The main reasons are as follows: (1) in the traditional nursing mode, because the diagnosis and treatment of each department is carried out independently, the departments cannot timely communicate the clinical diagnosis information of patients and cannot timely discuss the patient's condition, which may miss the best treatment time of patients, leading to increased difficulty in treatment. During the whole process, they can make clear their own division of labor and do their own work well in an orderly way and cooperate with the work of other departments, so as to develop the best and effective diagnosis and treatment plan for the treatment of patients and ensure the success rate of rescue [30]. (2) In addition, the traditional treatment mode only pays attention to the patient's body, but does not pay attention to the psychological status and needs of patients and their families, which cannot have a positive impact on the whole process of treatment. Therefore, a new, scientific, and effective emergency nursing mode is very important in the process of treatment of patients. In this study, nurses implemented targeted psychological intervention in patients during perioperative period, which effectively reduced the psychological stress reaction caused by patients' bad emotions and improved the treatment effect of patients [31]. (3) In this study, we consulted the most cutting-edge literature on emergency nursing at home and abroad in recent years and learned from the diagnosis and treatment experience of other major hospitals in this field. In the process of research and discussion, doctors of various departments expressed their opinions, so as to continuously optimize and improve the diagnosis and treatment plan. At the same time, with the help of the platform of multidisciplinary diagnosis and treatment mode, we finally determined the best treatment plan for patients, through the process of pre-examination, triage, and rescue, and the treatment effect of patients can be improved. (4) The research has multiple roles of multiple departments, which ensures that the operation of the organization is not affected by external factors and can be carried out smoothly in the process of treating patients. In this team, nurses carry out role coordination, establish the team supporting operation process and mechanism, formulate relevant standard system, train and assess team members, so as to ensure that all departments and roles can actively cooperate and assist, carry out standardized process implementation, and achieve better treatment effect. The emergency nursing mode constructed in this study is applied to the emergency treatment of patients with traumatic shock, which shortens the response time of hospital rescue, improves the success rate of rescue, reduces the incidence of complications, and improves the satisfaction of patients' family members [32]. On the one hand, the development of this study can provide a new idea for the first aid of patients with traumatic shock; on the other hand, it can also provide reference for the treatment of other diseases. However, due to time constraints, the sample size of patients included in the study is small, so it is necessary to expand the sample size in the future to further verify the effectiveness of the intervention program. At the same time, the process of emergency treatment of patients with traumatic shock also needs the active cooperation of various discipline teams, and the specific intervention plan should be summarized and further improved in practice [33]. Other studies have pointed out that when the body is seriously injured, it can cause acute circulatory insufficiency through vascular and nerve reflex and then lead to traumatic shock. The main clinical feature of the disease is microcirculation disorder, which can pose a greater threat to the life and health of patients. As a new nursing method, emergency nursing process can provide targeted nursing according to the actual situation of patients, and effectively shorten the treatment time through timely and accurate triage and reasonable arrangement of medical resources, so as to improve the success rate of rescue of patients to a large extent. In this study, the effective treatment time of the experimental group (emergency nursing mode) was shorter than that of the control group (routine emergency nursing), the rescue success rate of the experimental group was higher than that of the control group. The application of emergency nursing process can improve the rescue success rate of patients with traumatic shock, and shorten the effective treatment time. It is suggested to be popularized in clinical practice [34]. Foreign-related studies have pointed out that most of the trauma patients are caused by traffic accidents, high-altitude falls, and falls, which are sudden injuries. After admission, the patients should take timely hemostasis measures and give antishock treatment. In most cases, multidepartment consultation assistance is needed, and priority should be given to the treatment of fatal injuries. Under the premise of ensuring the stability of patients' vital signs, imaging scanning is carried out to make clear the location, degree, and nature of the injury, so as to formulate a targeted treatment plan. Most of the patients with acute trauma have serious injury, large amount of blood loss, and critical condition [35]. There are many patients with hemorrhagic shock. If effective treatment measures cannot be taken in time, they may die of excessive blood loss. The application of emergency nursing mode is to improve the quality of nursing. It requires the emergency department nurses to have higher and stronger comprehensive quality, so as to better perform the nursing task in the emergency care of patients with traumatic shock and to improve the work efficiency, information feedback, nursing quality of emergency medicine, equipment, personnel on duty, visiting, and triage; the transportation of the wounded has put forward higher requirements. The emergency nursing mode is also reflected in the integration and informatization, which can ensure the most timely and effective rescue of the critically ill while giving comprehensive first aid to the patients and improve the overall rescue success rate. The results showed that the effective rescue time of the observation group was significantly lower than that of the control group, and the rescue success rate and nursing satisfaction score of the observation group were significantly higher than those of the control group (*P* < 0.05). In short, the application effect of emergency nursing mode in patients with traumatic shock is significant, which can effectively improve the treatment efficiency and nursing satisfaction [36].

In this study, the rescue intervention, emergency stay, and preoperative preparation time of the study group were significantly shorter than those of the control group, the rescue success rate of 97.37% was significantly higher than that of 84.21% of the control group, the improvement rate of the study group was significantly higher than that of the control group, the disability rate was significantly lower than that of the control group, the overall emergency rescue effect was better than that of the control group, and the complication rate of the study group was 2.63% significantly lower than that of the control group (23.68%). The satisfaction rate of patients and their families in the study group was 97.37%, which was significantly higher than 84.21% in the control group (*P* < 0.05). It is suggested that the value of emergency nursing mode in the rescue of patients with traumatic shock is higher, which can fight for more time for surgery, improve the success rate and effect of rescue, and the safety and satisfaction are better than conventional rescue nursing.

## Figures and Tables

**Table 1:** Emergency intervention, emergency stay, and preoperative preparation time ($\bar{x}\pm s$).

Group	Time of emergency intervention (min)	Emergency stay (min)	Preoperative preparation time (min)
Control group (38)	14.00 ± 6.60	20.00 ± 4.00	13.70 ± 3.40
Study group (38)	8.30 ± 5.70	14.90 ± 4.20	10.30 ± 3.10
*t* value	4.029	5.420	4.555
*P* value	<0.001	<0.001	<0.001

**Table 2:** Rescue success rate (*n*)%.

Group	Number of successful rescue cases (*n*)	Rescue success rate (%)
Control group (38)	32	84.21
Study group (38)	37	97.37
*χ* ^2^ value	3.934	
*P* value	0.047	

**Table 3:** Emergency rescue effect (*n*)%.

Group	Improve (%)	Stable (%)	Permanent disability (%)
Control group (38)	15 (39.47)	18 (47.37)	5 (13.16)
Study group (38)	26 (68.42)	12 (31.58)	0 (0.00)
*χ* ^2^ value	6.408	1.983	5.352
*P* value	0.011	0.159	0.021

**Table 4:** Complications (*n*)%.

Group	Disseminated intravascular coagulation	Acute respiratory distress syndrome	Multiple organ dysfunction	Overall incidence (%)
Control group (38)	1	5	3	9 (23.68)
Study group (38)	0	1	0	1 (2.63)
*χ* ^2^ value	7.370			
*P* value	0.007			

**Table 5:** Satisfaction rate of patients and their families to rescue (*n*)%.

Group	Very satisfied	Quite satisfied	Not very satisfied	Satisfaction rate (%)
Control group (38)	29	3	6	32 (84.21)
Study group (38)	36	1	1	37 (97.37)
*χ* ^2^ value	3.934			
*P* value	0.047			

## Data Availability

The simulation experiment data used to support the findings of this study are available from the corresponding author upon request.
